This article has been retracted.

# Antimicrobial, antioxidant and cytotoxic properties of *Chenopodium glaucum* L.

**DOI:** 10.1371/journal.pone.0255502

**Published:** 2021-10-29

**Authors:** Safi Ullah Khan, Faizan Ullah, Sultan Mehmood, Shah Fahad, Arsalan Ahmad Rahi, Fayez Althobaiti, Eldessoky S. Dessoky, Shah Saud, Subhan Danish, Rahul Datta

**Affiliations:** 1 Department of Botany, University of Science and Technology Bannu, Bannu, KP, Pakistan; 2 Hainan Key Laboratory for Sustainable Utilization of Tropical Bioresource, College of Tropical Crops, Hainan University, Haikou Hainan, China; 3 Department of Agronomy, The University of Haripur, Haripur, Pakistan; 4 Department of Engineering, Faculty of Artificial Intelligence and Machine Learning, University of Hertfordshire, Hatfield, United Kingdom; 5 Department of Biotechnology, College of Science, Taif University, Taif, Saudi Arabia; 6 Department of Biology, College of Science, Taif University, Taif, Saudi Arabia; 7 Department of Horticulture, Northeast Agricultural University, Harbin, China; 8 Department of Soil Science, Faculty of Agricultural Sciences and Technology, Bahauddin Zakariya University, Multan, Punjab, Pakistan; 9 Faculty of Forestry and Wood Technology, Department of Geology and Pedology, Mendel University in Brno, Brno, Czech Republic; Harran Üniversitesi: Harran Universitesi, TURKEY

## Abstract

We evaluated phytochemical composition, antibacterial, antifungal, anti-oxidant and cytotoxic properties of aqueous (water) and organic extracts (methanol, ethyl acetate and *n*-hexane) of *Chenopodium glaucum*. Highest phenolic content 45 mg gallic acid equivalents (GAE)/g d.w was found in aqueous extract followed by ethyl acetate (41mg GAE/g d.w) and methanol extract (34.46 mg GAE/g d.w). Antibacterial potential of aqueous and organic extracts of *C*. *glaucum* was examined against *Acinetobacter baumannii*, *Klebsiella pneumoniae*, *Escherichia coli and Staphylococcus epidermidis*. The aqueous, methanolic, ethyl acetate, and *n*-hexane extract showed antibacterial activity against *A*. *baumannii*, *K*. *pneumoniae*, *E*. *coli and S*. *epidermidis*. However, against *A*. *baumannii* significantly higher inhibition zone (19 mm and 18.96 mm respectively) was shown by ethyl acetate and methanol extracts. Aqueous extract possessed highest growth inhibition (11 mm) against *E*. *coli*. Aqueous, ethyl acetate and methanol extracts showed 9 mm, 10 mm, and 10.33 mm zone of inhibition against the *K*. *pneumoniae*. For antifungal activity, the extracts were less effective against *Aspergillus niger* but showed strong antifungal activity against *Aspergillus flavus* (*A*. *flavus*). The antioxidant activity was measured as DPPH (2, 2-diphenyl-1-picrylhydrazyl), H_2_O_2_ and ABTS (2, 2’-azino-bis (3-ethylbenzothiazoline-6-sulfonic acid) scavenging activity of free radicals. All the organic extracts of *C*. *glaucum* possessed ABTS, DPPH and H_2_O_2_ scavenging properties. The highest cytotoxic activity measured as half maximal inhibitory concentration (IC50) against human lungs carcinoma cells was recorded for methanolic (IC50 = 16 μg/mL) and *n*-hexane (IC50 = 25 μg/mL) extracts, respectively. The Gas chromatography–mass spectrometry (GC-MS) analysis showed 4 major and 26 minor compounds in *n*-hexane extract and 4 major and 7 minor compounds in methanol extract of the *C*. *glaucum*. It is concluded that aqueous and organic extracts of *C*. *glaucum* would be potential therapeutic agents and could be exploited on a pilot scale to treat human pathogenic diseases.

## Introduction

Medicinal plants have been used by human beings in the treatment of pathogenic diseases since time immemorable. Presently approximately 80% of the population in developing countries use medicinal plants for the treatment of pathogenic diseases [1]. Roots, stem, leaves, and seeds of various plant species are reported to have antimicrobial and free radical scavenging properties [2] and used as natural antioxidants and antibiotics [3]. The greater use of medicinal plants in the treatment of pathogenic diseases is due to the fact that they are effective and safe, economical and usually have no side effects [4]. Medicinal plants have phytochemicals of biological significance and therapeutic value [5]. They contain natural antioxidants effective in the prevention of oxidative stress [6]. As a defense mechanism against pathogens and herbivores plants synthesize diverse groups of chemical compounds which can be used as alternatives to synthetic drugs [6]. The phytochemicals present in various organs of medicinal plants can be used as natural antioxidants, alternative to synthetic antibiotics, as food preservatives and nutraceuticals.

A large number of pathogenic bacterial and fungal species have been known to microbiologists. However, some of them are cosmopolitan and causative agents of severe human diseases. Bacterial species like *Escherichia coli* causes harmful diseases in human beings such as endemic problems, intestinal and extra intestinal problems [7]. The *Acinetobacter baumannii* is an opportunistic pathogen and causes infection in lungs, blood and urinary tract [8]. The *Klebsiella pneumoniae* causes different infections like pneumonia, urinary tract infections, diarrhea, upper respiratory tract infection, meningitis and wound infection [9]. The *Staphylococcus epidermidis* is the cause of various infections, especially as a biofilm on surgical devices [10]. Fungal species such as *A*. *niger* causes otomycosis [11] and cutaneous infections [12]. Moreover, there are reports of *A*. *niger* causing pneumonia and other pulmonary infections [12]. The *A*. *flavus* causes aspergillosis diseases in immune compromised persons. Moreover, it is a major producer of aflatoxin a potent carcinogen [13].

Recently synthetic antibiotics are extensively used in the treatment of human diseases caused by diverse groups of pathogens. However, studies have indicated that bacterial and fungal strains can gain resistance to synthetic antibiotics [14,15]. Therefore, plant-derived compounds in the treatments of pathogenic diseases offer a plausible option [16]. Various studies have reported the use of plants extracts as antibacterial, antifungal, anti-oxidative, and anticancer agents [17].

Cancer is among the leading causes of death across the globe such that 1 in 6 deaths is caused by cancer. Nearly 70% of deaths caused by cancer are reported in middle and low-income countries [18]. Lung cancer, blood cancer, prostate cancer, breast cancer and cervix cancer are the most common types of cancer found in human population globally. Cancer is a cluster of diseases caused due to loss of genetic control on cell cycle which results in uncontrolled and abnormal cell growth [19]. Treatment of cancer is very expensive in developing countries. The conventional methods like chemotherapy, surgery, hormone therapy and radiotherapy are commonly used in the treatment of cancer. However, these conventional methods of cancer treatment have been associated with severe side effects [20]. This has led scientific community for searching more effective and new drugs with minimum side effects [21]. Phytochemicals and natural antioxidants found in plants have been reported for their pro-apoptotic and anti-proliferative properties. Out of 200 chemical compounds approved for the treatment of cancer, 50% of that are derived from natural products [22].

*Chenopodium glaucum* belongs to the family Chenopodiaceae. It is a small annual herb having flashy leaves widely distributed in Europe, Central and Eastern Asia, North America, and Australia. It preferably grows along roadsides, gardens, and lake shores. Some allied species of *C*. *gluaccum* are found in South Africa, North America, and New Zealand (http://www.tropicos.org/Project/Pakistan). Several members of the genus *Chenopodium* are highly medicinal exhibiting antibacterial, antifungal, anti-diaphoretic and anti-asthmatic properties [23,24].

Scientists are always interested in the extraction and characterization of biologically active components from medicinal plants. Then these compounds are tested for antimicrobial, antioxidant and anticancer properties. Moreover, attention is also paid to link modern scientific evidences with traditional therapeutic system. The people in Pakistan have been using many plant species as traditional medicines, but there has been a lack of sufficient data about their *in vitro* and *in vivo* efficacy using modern scientific approaches. Therefore, in the present studies, we have tested and compared aqueous and organic extracts of *C*. *glaucum* for antimicrobial, antioxidant, and cytotoxic properties using modern scientific techniques.

## Materials and methods

The *C*. *glaucum* specimens were collected from Mama Khel of District Bannu, Pakistan, and identified by Dr. Faizan Ullah Department of Botany University of Science and Technology Bannu. The specimen of *C*. *glaucum* was prepared and stored in the herbarium for future reference (voucher No. Cg-C-1). The above ground parts of 100 plants were collected, washed with tap water, and dried for three weeks in the shade. The plant material was ground to a fine powder with an electric grinder. The ground plant material (50 g) was extracted separately in methanol, water, ethyl acetate and *n-*hexane for 48 hours at room temperature. The extracts were then filtered using Whatman No.1 filter paper. The extracts were then dried by evaporating solvents in a rotary evaporator (Model, RE301, Japan) Thick, gummy extracts obtained were collected in small vials and stored at 4°C in a refrigerator.

### Total phenolic contents

Swain and Hillis method [25] was followed to determine soluble phenolics content of *C*. *glaucum*. The 1 mg/mL of the methanol, ethyl acetate, *n-*hexane, and aqueous extracts were prepared in respective solvents. A 250 μL of the extracts were mixed with Folin-Ciocalteau reagent (250 μL) and an aqueous sodium carbonate solution (7.5%). Reaction mixtures were kept in the dark for one hour at 25°C. The absorbance was measured at 765nm using a spectrophotometer (SP-3 Tokyo, Japan). Different concentrations (0–32 μg) of gallic acid (GAE) solutions were prepared for standard curve formation. The concentration of total phenolics compounds was expressed as mg GAE equivalents/g extract.

### Antibacterial activity

Agar well diffusion method was followed for antibacterial tests [26]. Agar medium was prepared by dissolving 28g of agar in 1L of distilled water and sterilized in an autoclave at 121°C for 20 minutes. The melted agar was poured into sterile Petri dishes (25 cm) and allowed to solidify. Five wells of 3 mm diameter were aseptically punched on agar plates using a sterile cork borer. The extract (30 mg) was dissolved separately in 1ml dimethyl sulfoxide (DMSO). Fixed volume (0.1ml) of all the extracts was introduced in four peripheral wells and a central well with standard (streptomycin). Fresh bacterial strains (*Acinetobacter baumannii*, *Staphylococcus epidermidis*, *Escherichia coli* and *Klebsiella pneumoniae*) were swabbed on the Petri dishes separately. The Petri dishes were placed in an oven at 38°C for 28 hours. Antibacterial tests of the extracts against the test bacterial strains were represented by growth free zone of inhibition (mm) near each well.

### Antifungal activity

Antifungal activity of the crude extracts was determined according to the method of Choudhary et al. [27]. Sabouraud dextrose agar (Merck, Darmstadt, Germany) was used for inoculum preparation of the fungal strains. 200μg/ml of the final concentration was prepared from the initial stock of 12mg/ml for antifungal activity. The terbinafine solution prepared in DMSO (12 mg/ml) was used as a positive control, whereas the negative control had only pure DMSO. The SDA media and test tube sterilization were made at 121°C for 20 minutes. The test tubes containing media were solidified in a slant position. One-week old culture of *A*. *Niger* and *A*. *flavus* were used for inoculation.

The control (positive and negative) test tubes were also added with DMSO and terbinafine, respectively. The test tubes were kept in an incubator at 28°C for seven d. In all the test tubes, the linear growth of fungi was measured in mm. The inhibition in fungal growth was noted by comparing it with negative control. Inhibition of fungal growth was determined using the following equation

$$Fungal\;growth\;inhibition\;\left(\%\right)=100\left[\frac{\left(linear\;growth\;in\;test\;sample\;in\;mm\right)}{\left(linear\;growth\;in\;control\;mm\right)}\right]\times 100$$

### ABTS scavenging activity

ABTS scavenging activity was performed according to method of Re et al. [28]. The 7mM ABTS solution was prepared by dissolving 0.32g of ABTS in 83ml of distilled water. A 2.45 mM potassium per sulfate solution was prepared by dissolving 0.22g of potassium persulphate in 0.3L of distilled water. ABTS free radical was produced by mixing of 7mM ABTS and 2.45mm of potassium per sulphate in the equal ratio (1:1). The mixture was placed in darkness for 12–16 hours at 25°C. ABTS solution was diluted with methanol, and the absorbance of the solution was adjusted to 0.700 at 734nm. A 5μl of each of the extract was added in 3.995 ml of diluted ABTS^+^ radical solution. The absorbance was taken at 734nm and % inhibition was calculated using the following formula.


$$\mathrm{Inhibition}\;\left(\%\right)=\frac{\mathrm{Ac}-\mathrm{As}}{\mathrm{Ac}}\times 100$$

Ac = control absorbance, As = sample absorbance. Ascorbic acid was considered as a standard substance.

### DPPH scavenging activity

Brand-Williams et al. [29] protocol was followed to determine antioxidant capacity by DPPH (1, 1, biphenyl, 2-picrylhydrazyl) test. 2.4 mg of DPPH was dissolved in 100 ml of methanol. 5μl of the different extracts was added to 4 ml of Methanolic DPPH. The reaction mixture was shaken and kept at 25 degrees centigrade in the dark for 30 min. Reading of the reaction mixture was taken at 515 nm through a spectrophotometer. Percentage inhibition was taken using the following formula.

$$\mathrm{DPPH}\;\mathrm{Scavenging}\;(\%)=\frac{\left(\mathrm{Blank}\;\mathrm{absorbance}-\mathrm{sample}\;\mathrm{absorbance}\right)}{\left(\mathrm{Blank}\;\mathrm{absorbance}\right)}\times 100$$

where, the absorbance of blank at t = 0 min; absorbance of the mixture at t = 30 min.

### Hydrogen peroxide scavenging activity

Hydrogen peroxide scavenging activity was performed according to the method of Ruch et al. [30]. A phosphate buffer of 7.4 pH was used for the preparation of Hydrogen peroxide solution (40mM). 100 μg/ml solution of each aqueous, ethyl acetate, methanol, and hexane were prepared in distilled water. 0.6 ml of each of these extracts was added to H_2_O_2_ solution.

10 min after preparation of the extract, absorbance at 230nm was taken. Phosphate buffer without hydrogen peroxide was taken as a blank. The scavenging of H_2_O_2_ (%) was taken as:

$$Scavenged\;\left[H_{2}O_{2}\right]\;\left(\%\right)=\left[\left(AC–AS\right)/AC\right]\times 100$$

Where AC = Control absorbance, AS absorbance at the presence of the sample, Ascorbic acid was taken as a standard antioxidant.

### Cytotoxicity assay

The procedure for the evaluation of cytotoxicity initially determines the potential of already cultured cells to multiply in the existence of a test compound and then quantify total protein concentration using sulforhodamine B dye to determine living cells percentage. The cytotoxic property of aqueous and organic extracts of *C*. *glaucum* was checked on the human lung carcinoma (LU-1) at 1–48μg/mL in dimethyl sulfoxide. Cell cultures as 3 x 10^5^ cells/mL were grown in ninety-six wells plate and test samples (10 μL) were put into each and every well. Incubation of plates was performed in an incubator (Biotech) in the presence of humidified air with CO_2_ (5%) at 37°C. Cell viability test was performed with SRB staining technique [31]. The half maximal inhibitory concentration (IC50 values) was recorded as the concentration of testing compound effective in inhibiting cell growth by 50%. HPLC grade Colchicine (Sigma Aldrich, USA) was used and kept as a positive control whereas, 0.5% DMSO was used as a negative control.

### GC-MS procedure

The GC-MS analysis of methanol and *n*-hexane extracts was done on a GCMS-QP 2010 Plus fixed was Rtx-5MS capillary column (30 m × 0.25 mm internal diameter, 0.25 μm film thickness: maximum temperature, 350°C). The carrier gas used was ultra-pure helium (99.99%) with a 1.2 mL/min flow rate. The oven temperature was set constant at 80°C- 220°C as 5˚C/min. The crude extracts were diluted with respective solvents (1/100 v/v %) and then filtered. Clear filtered extracts as 1 μL were injected into the injector with a split ratio of 30:1. Full-scan mass spectra in a range of 40–550 amu were obtained. The bio compounds present in extracts were taken in percentage by peak area measurement and retention time. The mass spectra matching was done with those of already available spectra of standards in mass spectrum library. The names, molecular weights, and structures of the compounds in extracts were ascertained.

### Statistical analysis

In this study mean values of the different biological assays were analyzed via one way Analysis of Variance (ANOVA). Significant differences among mean values were calculated at p < 0.05 by using least significant difference test [32]. In order to calculate IC_50_ values linear regression analysis was performed.

## Results

### Total phenolics

The total soluble phenolic content of *C*. *glaucum* was determined in aqueous, ethyl acetate, methanol, and *n*-hexane extract (Fig 1). The highest phenolic content (45 mg GAE/g d.w) was found in an aqueous extract prepared, followed by ethyl acetate (41 mg GAE/g d.w) and methanol extract (34.46 mg GAE/g d.w) and the lowest recorded in *n*-hexane extract (24.57mg GAE/g d.w).

**Fig 1:** Total phenolics content of aqueous, methanol, hexane, and ethyl acetate extracts of *C*. *glaucum*.

### Antibacterial activity

We found that various organic extracts of *C*. *glaucum* exhibited antibacterial activity against the tested bacterial strains (Fig 2). Highest zone of inhibition (19 mm and 18.96 mm) against *A*. *baumannii* was shown by ethyl acetate and methanol extracts, respectively. Aqueous extract possessed higher growth inhibition (11 mm) against *E*. *coli*. The *n-*hexane, ethyl acetate, and methanol extracts have statistically similar antibacterial activity and lower (10%) than aqueous extract against *E*. *coli*. Against the *K*. *pneumoniae*, aqueous, ethyl acetate, and methanol extracts have a similar zone of inhibition (9, 10, 10.33 mm), which was higher (<44%) than ethyl acetate extract. Significantly higher (p<0.05), the aqueous extract showed antibacterial activity. The aqueous extract resulted in 11 mm zone of inhibition. The *n*-hexane, ethyl acetate, and methanol extracts showed 9 mm, 10 mm, and 6mm zone of inhibition, respectively, against *S*. *epidermidis*.

**Fig 2:** Antibacterial activity of aqueous, methanol, hexane and ethyl acetate extracts of *C*. *glaucum* on different strains of bacteria.

### Antifungal activity

The anti-fungal activity of aqueous, *n-*hexane, ethyl acetate, and methanol extract was determined against 2 different fungi species (Fig 3). The result of the fungi’s linear growth in the extract was compared with the standard drug, terbinafine. The extracts showed weak antifungal activity against *A*. *niger* (approximately 19%), while strong antifungal activity against *A*. *flavus* (about 57%). From the above results, it is clear that *A*. *niger* is resistant to the extracts of *C*. *glaucum*. Whereas *A*. *flavus* is susceptible to these extracts.

**Fig 3:** Antifungal activity of aqueous, methanol, hexane and ethyl acetate extracts of *C*. *glaucum* on two different strains of fungi.

### 2, 2-azinobis (3-ethylbenzo-thiazoline-6-sulfonate) ABTS* scavenging ability

Percent scavenging effect of ABTS in aqueous, methanolic, ethyl acetate, and *n-*hexane extracts of *C*. *glaucum* is shown in Fig 4. The highest antioxidant activity (83%) was recorded for aqueous extract at 300 μg/ml. Ethyl acetate and methanol extracts at this concentration also showed high antioxidant activity (82%) next to aqueous extract. The *n*-hexane extract showed the lowest antioxidant activity (75%) among the four tested extracts.

**Fig 4:** The ABTS scavenging activity of aqueous, methanol, hexane, and ethyl acetate extracts of *C*. *glaucum*.

### DPPH free radical scavenging activity

The aqueous and methanolic extracts at all the three concentrations (300, 150, and 75 μg/ml) showed high free radical scavenging activity; however, maximum (60% and 59% respectively) DPPH free radicals scavenging activity of the two extracts were recorded at 300 μg/ml. At 300 μg/ml ethyl acetate and *n-*hexane extracts showed 58% and 56% DPPH free radicals scavenging activity (Fig 5).

**Fig 5:** The DPPH scavenging activity of aqueous, methanol, hexane and ethyl acetate extracts of *C*. *glaucum*.

### Hydrogen peroxide scavenging capacity

The hydrogen peroxide scavenging capacity of aqueous, *n*-hexane, ethyl acetate, and methanol extracts are given in Fig 6 and compared with ascorbic acid as standard. The antioxidant activity of the extract is high in higher concentrations of each extract. The aqueous and methanol extract of *C*. *glaucum* showed a high degree of antioxidant activity (70%) as compared to ethyl acetate and hexane extract (68% and 67%) respectively at 300 μg/ml.

**Fig 6:** H_2_O_2_ scavenging activity of aqueous, methanol, hexane, and ethyl acetate extracts of *C*. *glaucum*.

### Cytotoxic activity

We found a concentration-dependent inhibitory effect of the extracts on the human lung carcinoma cells (Fig 7). Methanol extract showed the most substantial inhibitory effect on human lung carcinoma cells (IC50 = 16 μg/mL) followed by *n*-hexane extract (IC50 = 25 μg/mL). The lowest inhibitory effect on human lung carcinoma cells was shown by ethyl acetate extract (IC50 = 55 μg/mL).

**Fig 7:** Cytotoxicity of *C*. *glaucum* extracts against human lung carcinoma cells.

### GC-MS analysis

The GC-MS analysis of *n*-hexane and methanol extracts showed diverse groups of phytochemicals (Tables 1 and 2). Some compounds like phytol, Pentadecanoic acid, 14 methyl-, methyl ester, and beta-Ionone were present in both extracts. However, phytol concentration (39.49%) and Pentadecanoic acid, 14 methyl-methyl ester (15.49%) were higher in *n*-hexane extracts than that of methanol extract. Major phytochemicals in methanol extract were Chloroacetic acid, 2-pentyl ester (56.21%) followed by 3-Hexane-2-one, 3,4-dimethyl-,(Z)- (10.6%), Linolelaidic acid, methyl ester (7.1%), and Aromadendrene (5.55%). In *n*-hexane extract next to phytol and Pentadecanoic acid, 14 methyl-methyl ester other major constituents were 9,12-Octadecadienoyl chloride, (Z,Z)-(13.14%) and (3,3-Diflouro-2-propenyl) (trimethyl) silane (5.13%).

**Table 1:** Bioactive compounds in *n*-hexane crude extract.

S/No	Compound name	Molecular formula	Retention time	Concentration (%)
1	Phytol	C_20_H_40_O	28.350	39.49
2	Pentadecanoic acid, 14 methyl-,methyl ester	C_17_H_34_O_2_	24.760	15.49
3	9,12-Octadecadienoyl chloride, (Z,Z)-	C_18_H_31_ClO	28.107	13.14
4	(3,3-Diflouro-2-propenyl)(trimethyl)silane	C_6_H_12_F_2_Si	11.186	5.13
5	9,12-Octadecadienoic acid,methyl ester, (E,E)-	C_18_H_32_O_2_	27.984	3.62
6	Decane	C₁₀H₂₂	5.991	2.48
7	Dihydroactinidiolide	C_11_H_16_O_2_	16.249	2.21
8	2-Phenyldodecane	C18H30	22.351	1.98
9	Octanal,7-methoxy-3,7-dimethyl-	C_11_H_22_O_2_	28.927	1.67
10	Tetrahydrogeranylacetone	C_13_H_22_O	23.136	1.60
11	4-Phenyldodecane	C_18_H_30_	18.858	1.31
12	Hexadecylene oxide	C_16_H_34_	23.034	1.16
13	1-Iodo-2-methylnonane	C_10_H2_1I_	17.838	1.16
14	6-Phenyldodecane	C_18_H_30_	20.721	0.97
15	Tridecane	C_13_H_28_	8.180	0.94
16	3-Phenyldodecane	C_18_H_30_	21.544	0.93
17	5-phenyleicosane	C_26_H_46_	20.822	0.91
18	Dichloroacetic acid, 4-pentadecyl ester	C_17_H_33_ClO_2_	26.098	0.78
19	Undecane,2,8-dimethyl-	C_12_H_26_	26.2200	0.78
20	Hexadecane	** **C_16_H_34_	22.206	0.77
21	(1-Ethylundecyl)benzene	C_19_H_32_	23.684	0.63
22	1-Dodecene	C_12_H_24_	22.060	0.57
23	Pentaflouropropionic acid, dodecyl ester	C_15_H_25_F_5_O_2_	17.631	0.56
24	Tridecane	C_13_H_28_	24.257	0.54
25	Z-4-Octadecan-1-ol acetate	C_20_H_38_O_2_	23.909	0.44
26	beta-Ionone	C_13_H_20_O	15.191	0.44
27	Undecane	C_11_H_24_	13.048	0.41
28	6,10-Dodecadien-1-yn-3-ol,3,7,11-trimethyl-	C_15_H_24_O	24.632	0.28
29	Isooctanol	C_8_H_18_O	12.846	0.20
30	(2E)-3,7,11,15-Tetramethyl-2-hexadecen-1-ol	C_20_H_40_O	23.540	0.19

**Table 2:** Bioactive compounds in methanolic crude extract.

S/No	Compound name	Molecular formula	Retention time	Concentration (%)
1	Chloroacetic acid,2-pentyl ester	C_7_H_13_ClO_2_	5.853	56.21
2	3-Hexane-2-one,3,4-dimethyl-,(Z)-	C_8_H_14_O	11.879	10.69
3	Linolelaidic acid,methyl ester	C_19_H_32_O_2_	27.981	7.10
4	Aromadendrene	C_19_H_32_O_2_	13.713	6.51
5	1,5,9,11-Tridecatetraene,12-methyl-,(E,E)-	C_14_H_22_	17.588	5.55
6	Pentadecanoic acid,14-methyl-,methyl ester	C_17_H_34_O_2_	24.758	4.86
7	Hexadecanoic acid,15-methyl-,methyl ester	C_18_H_36_O_2_	28.593	4.40
8	Phytol	C_20_H_40_O	28.339	2.34
9	9,12-Octadecadienoyl chloride,(Z,Z)-	C_18_H_31_ClO	28.101	1.82
10	beta-Ionone	C_13_H_20_O	15.200	0.27
11	Tetrahydrogeranylacetone	C_13_H_22_O	23.137	0.25

## Discussion

Plants are potential sources of therapeutic agents. Traditional use of plants extract has been very ancient in treating viral, fungal, bacterial, and other microbial diseases [33]. The present study results revealed that ethyl acetate and methanolic extracts of *C*. *glaucum* have a higher growth inhibitory effect on *A*. *bauminni*, aqueous extract on *E*. *coli*, aqueous, ethyl acetate, and methanol extracts on *K*. *pneumoniae*, and aqueous and ethyl acetate extracts on *S*. *epidermidis*. Other species of the genus Chenpodium like *Chenopodium ambrosioides* and *Chenopidium album* have been reported for antibacterial properties [34,35]. The variations in the efficacy of different plant extracts as antibacterial agents may be because of their composition of biologically active compounds [36]. Octadeconoic acid found in methanolic extract has been reported for antimicrobial properties [37].

The aqueous extract of *C*. *glaucum* showed higher antifungal activity against *A*. *niger* and *A*. *flavus* compared to methanol, ethyl acetate, and *n-*hexane extracts. From the above results, it is clear that *A*. *niger* is resistive to the extracts of *C*. *glaucum* and *A*. *flavus* is susceptible to these concentrations of extracts. Aqueous extract of plant species like Juglan spp. and Solanum spp. have been reported to show strong antifungal activity against fungal pathogens due to their higher phenolics content [38]. The higher antimicrobial activity can be due to the high concentration of phenolic compounds in aqueous, ethyl acetate, and methanolic extracts. In the present study, we found that aqueous extract possessed the highest amount of phenolic compounds compared to ethyl acetate, methanol, and *n-*hexane extracts making it highly antimicrobial. Ozsoy et al. [39] have mentioned higher concentration of phenolics in aqueous extract of *Smilax excels*. Variations in phenolics content of various extracts may be attributed to the solvents’ polarity such that polar solvents extract more phenolics as compared to non-polar extracts [40]. Similar results are reported by Lee et al. [41] that water is the most suitable solvent for the extraction of phenolics from plant parts. Pervez et al. [42] also mentioned the higher amount of phenolics in water extract of *Moringa oleifera*. The mechanism involved in antimicrobial activity is the cytoplasm granulation, cell membrane rupture, inhibition of enzymes involving cell wall, protein, amino acid synthesis, and sphinophspholipid biosynthesis and electron transport chain [43].

Our research work showed that whole-plant extracts of *C*. *glaucum* exhibited antioxidant properties measured as ABTS, DPPH and Hydrogen per oxide scavenging activity. The difference in antioxidant properties of different extracts may be due to the polarity of the solvents used in the study as highly polar solvents have greater potential for the extraction of phenolic compounds, which are strong antioxidants [44]. Hajji et al. [45] reported that aqueous extract of Mirabilis possessed significant free radical scavenging activity. Literature also reports the correlation of a plant extract’s total phenolics with its antioxidant activity [46,47]. Like aqueous extract, *n*-hexane and methanolic extracts also exhibited antioxidant properties which might be due to the presence of compounds like Phytol, Pentadecanoic acid, 14 methyl-,methyl ester, Dihydroactinidiolide, 9,12-Octadecadienoyl chloride,(Z,Z)-, Aromadendrene, Pentadecanoic acid,14-methyl-, methyl ester, 9,12-octadecadienoicacid (Z,Z)-, methylester, 9,12-Octadecadienoyl chloride,(Z,Z)- which have been reported for strong antioxidant properties [48–51].

We observed that methanolic and *n*-hexane extracts were highly cytotoxic on human lungs carcinoma cells. Some of the phytochemicals present in *n*-hexane and methanolic extracts have proven pharmacological significance. We found that phytol was present in both extracts. Phytol has been reported as a potent antimicrobial, antioxidant and anticancer agent [50]. Moreover, phytol is an essential precursor for vitamin K and E and has been proven to possess cytotoxic properties against breast cancer cell lines [52,53]. Aromadendrene found in the methanolic extract is reported to induce apoptosis in skin epidermoid cancer cells [54]. Our study documents the first-time anticancer properties of *C*. *glaucum*. This study also suggests that apart from phenolic compounds, other compounds found in methanolic, and *n*-hexane extracts also possess strong anticancer activity.

## Conclusions

This study showed that *C*. *glaucum* extracts have antimicrobial, antioxidant, and anticancer properties. Aqueous and methanolic extracts were powerful antimicrobial agents. However, the higher anticancer property was recorded for methanolic and *n*-hexane extracts. Biological activities of *C*. *glaucum* are credited to the presence of diverse groups of compounds in different extracts. Overall, this study provides bases for further clinical trials focusing on antioxidant and chemotherapeutic properties of *C*. *glaucum*.
